The article "The Studies of Chlorogenic Acid Antitumor Mechanism by Gene Chip Detection: The Immune Pathway Gene Expression" was retracted in 2020. Reason: no approval from a third party.

# The Studies of Chlorogenic Acid Antitumor Mechanism by Gene Chip Detection: The Immune Pathway Gene Expression

**DOI:** 10.1155/2013/617243

**Published:** 2013-05-09

**Authors:** Tian Yi Kang, Hua Rong Yang, Jie Zhang, Dan Li, Jie Lin, Li Wang, XiaoPing Xu

**Affiliations:** ^1^West China School of Pharmacy, Sichuan University, Chengdu 610041, Sichuan Province, China; ^2^Jiuzhang Biochemical Engineering Science and Technology Development Co., Ltd, Chengdu 610041, Sichuan Province, China

## Abstract

Persistently increasing incident of cancer in human beings has served to emphasize the importance of studies on mechanism of antitumor substances. Chlorogenic acid (CA), extracted from folium cortex eucommiae, has been confirmed to have lots of biological activities encompassing inhibition of tumor. However, the anticancer mechanism of CA remains unclear. Here, we have utilized a whole mouse genome oligo microarray (4∗44K) to analyze gene expression level of female BALB/c mice (implanted with EMT-6 sarcoma cells) after treatment with low, medium, and high-dose CA (5 mg/kg, 10 mg/kg, and 20 mg/kg), docetaxel, interferon, and normal saline separately at 6 time points (3rd, 6th, 9th, 12th, 15th, and 18th days after administration). Differentially expressed genes screened out by time-series analysis, GO analysis, and pathway analysis, and four immune-related genes were selected for further confirmation using RT-qPCR. The results demonstrated that CA is able to change gene expression and that the responsive genes (CaN, NFATC2, NFATC2ip, and NFATC3) involved in immune pathways had been significantly upregulated by CA. Expression of immune factors such as IL-2R and IFN-**γ** can be improved by CA to promote activation and proliferation of T cells, macrophages, and NK cells, thus enhancing their surveillance and killing abilities, further suppressing the growth rate of tumor cells.

## 1. Introduction

Cancer dormant cell theory takes the view that activation of resting cells is the key factor causing cancer metastasis. Recent studies indicate that resting cells can be activated through escaping immune surveillance when immune function is weakened and that energy used for cell revivals can be provided by the newborn vessels [1–3]. Therefore, the study on improving body immune surveillance and restraining the energy of tumor growth will be an emergent mission as well as a breakthrough in the field of clinical treatment of cancer. 

Chlorogenic acid (CA), extracted from folium cortex eucommiae and the flower bud of* Lonicera confusa*, is a kind of depside formed by caffeic acid and quinic acid. A large number of studies on CA have demonstrated that CA has a wide range of biological activities including inhibition of tumor cells [4]. According to preliminary studies, we recognize that CA is able to inhibit tumor in mouse except for these with T-cells defect, which suggests that immune system can be one of the targets of tumor suppression. Meanwhile, *in vivo* studies of our group indicate that CA also changes the advantage state of Th2 drift of BALB/c EMT-6 mice. It significantly enhance the activities of BALB/c EMT-6 mice cytotoxic T lymphocyte and natural killer cells as well as strengthening macrophage phagocytosis activity and lymphocyte transcription activity, thus boosting specific and nonspecific cellular immune function to tumor cells. Recent studies show that antitumor property of CA may have a connection with its ability of enhancing the activities of aryl hydrocarbon hydroxylase, suppressing formation of 8-OH-dG, carcinogen-DNA adduct, and oxygen radical [5, 6]. Meanwhile, CA can guard against gastric cancer and colon cancer and even suppress related carcinogenic factors [7, 8]. *In vitro* studies revealed that CA can enhance T-cell proliferation caused by influenza virus antigen and can induce the generation of IFN-*γ* and IFN-*α* by human lymphocytes and peripheral blood leukocytes [9, 10]. Additionally, we find that CA can also activate neurocalcin to strengthen the activity of macrophagocyte [11]. Although much evidence has proved the anticancer property of CA, little is known about its exact targets on molecular level.

The article "The Studies of Chlorogenic Acid Antitumor Mechanism by Gene Chip Detection: The Immune Pathway Gene Expression" was retracted in 2020. Reason: no approval from a third party.

Base on the principle of complementary base pairing, microarray technology can distinguish particular genes from the mixture of genes by taking advantage of gene probes. Different from normal PCR, RT-qPCR can take quantitative analysis of unknown system. Meanwhile, its sensitivity, accuracy, and specificity are better than those of normal PCR. To explore the expression level of genes in tumor cells, we utilized a microarray technique to detect BALB/c EMT-6 mice after treatment with CA, docetaxel, interferon, normal saline separately, and the differences in expression level were confirmed by RT-qPCR. Time-series analysis, GO analysis, and pathway analysis were used to screen out common genes and analyze the relationship between putative genes and anticancer process of CA. Our data has suggested that CA is able to inhibit the growth of tumor through regulating immune system.

## 2. Materials and Methods

### 2.1. Animal Model Construction and CA Treatment

Female SPF mice (BALB/c) used in this experiment weigh 17-18 g on average, provided by the animal center of Sichuan University. EMT-6 sarcoma cells were provided by West China Hospital of Sichuan University Department of Health Engineering Key Laboratory of Transplantation and Transplantation Immunity.

The article "The Studies of Chlorogenic Acid Antitumor Mechanism by Gene Chip Detection: The Immune Pathway Gene Expression" was retracted in 2020. Reason: no approval from a third party.

We took EMT-6 cell line out of the −152°C ultra low temperature refrigerator. After thawing, centrifuging, and primary culturing, we used 0.25% trypsin for digestion twice and then subcultured it to a required number. All the collected cells were diluted with phosphate-buffered saline (PBS) in the end. Each BALB/c mouse was injected with 0.2 mL cell solution. The tumor would not transfer until it grew to a certain size. We homogenized the tumor taken from the body of BALB/c tumor-bearing mice to cell suspension and then inoculated the cell suspension to other BALB/c mice. Mice used for microarray analysis were injected with high-dose CA (experimental group), docetaxel (control group), and normal saline (negative control group). Gene expression of experimental group was analyzed at six time points (3rd, 6th, 9th, 12th, 15th, and 18th days, resp., after administration), while the control group and negative control group were both analyzed at the 12th days after administration. RT-qPCR took mice injected with low, medium, and high-dose CA (5 mg/kg, 10 mg/kg, 20 mg/kg) as experimental group, docetaxel and interferon as control group, and normal saline as negative control group. Each of these groups was tested 12 days after administration.

### 2.2. RNA Extraction and Labeling

Total RNA was extracted using mirVana RNA Isolation Kit (Applied Biosystem p/n AM1556) in 15 min after tissue collection. Quality and concentration of RNA were checked by spectrophotometer analysis and gel electrophoresis. All extracted samples had an A260/280 ratio of between 2.0 and 2.1 and a 28S/18S ratio of 2 [12]. Agilent 2100 Bioanalyzer was used for further verification and qualified RNA had an RIN greater than 7.0. Total RNA was transcribed to double-stranded cDNA using RevertAid First Strand cDNA Synthesis Kit (Fermentas), with T7 Promoter Primer. The aaUTP-labeled cRNA was produced from cDNA by *in vitro* transcription. cRNA was dyed with Cy3 and purified using RNeasy Mini Kit (Qiagen, Valencia, CA, USA) according to the protocol of the RNeasy Plus Mini Kit.

### 2.3. Hybridization and Scanning

Cy3 cRNA must be fragmented in a buffer of 11 *μ*L 10× blocking agent, 2.2 *μ*L 25× fragmentation buffer and a certain amount of nuclease-free water at 60°C for half an hour before hybridization. We added 55 *μ*L 2× GEx hybridization buffer to the denatured and fragmented cRNA and then transfered them to microarrays at 65°C for 17 h with constant rotation. After hybridization, the microarrays were washed twice with buffer 1 for 1 minute followed by buffer 2 at 37°C for 1 minute too. In the end, the microarrays were autoscanned twice in 100% and 10% PMT, respectively, at 5 *μ*m resolution. The data was analyzed by Agilent Feature Extraction software and the quantile normalization was finished by GeneSpring 10.0.

The article "The Studies of Chlorogenic Acid Antitumor Mechanism by Gene Chip Detection: The Immune Pathway Gene Expression" was retracted in 2020. Reason: no approval from a third party.

### 2.4. Microarray Data Preprocessing

After acquisition of raw data, Agilent Feature Extraction software kit was used to eliminate the effect of background signals through automatic gridding. We took the log 2 of the normalized background adjusted values to narrow the threshold of fluorescence signal strength before quantile normalization by GeneSpring 10.0 and then used a linear model to estimate expression values on the log scale. Both programs were available in the limma package. We chose a standard among the microarray samples thus the whole microarray data varied on it to obtain the same baseline of average density. Unqualified probes should be filtered out. Differentially expressed genes are submitted to Student's *t*-test and *P* ≤ 0.05.

### 2.5. Interaction Network Analysis

We inputted the data of probes used for gene expressing analysis into SBC Analysis System (V2010.05).

### 2.6. RT-qPCR

RNA extracted from experimental group of CA, positive control group of docetaxel, and interferon, negative control group were used to measure expression of selected genes of interest by RT-qPCR. Genes CaN, Nfatc2, Nfatc3, and Nfatc2ip showed a different expression level following treatment with low, medium, and high-dose CA, respectively. Primers used for RT-qPCR validation were designed according to each gene sequence and finished by SBC. Primer names, accession numbers, and sequences are listed in Table 1. 

Total RNA was isolated using TRIzol reagents. The RNA integrity was verified with RNA formaldehyde electrophoresis and the quality was detected by spectrophotometry. The RNA samples had an A260/280 ratio of greater than 2 and a 20sRNA/18sRNA ratio of greater than 1.1. Single strand cDNA was synthesized using RevertAid First strand cDNA Synthesis Kit. Reverse transcription reactions were conducted at 42°C for 30 min and at 85°C for 5 min at a 20 *μ*L total reaction volume containing the following reagents: 2 *μ*L RNA, 1 *μ*L oligo, 2 *μ*L (10 mM) dNTP mixture, 1 *μ*L RiboLock RNase Inhibitor, 4 *μ*L 5× reaction buffer, 9 *μ*L water, and 1 *μ*L RevertAid M-MuLV. PCR was performed using a Sino Bio Taq 2× Master Mix. The RT-qPCR products were analyzed by 1.0% agarose gel electrophoresis.

PCR reaction should be taken at a temperature gradient in the range of annealing temperature of CaN, Nfatc2, Nfatc3, and Nfatc2ip. RT-qPCR analysis was conducted to obtain crossing point (Ct) values of each gene and standard curve was established through the linearity between Ct value and log 2 of expression values. Before carrying out RT-qPCR analysis, cDNA and primers should be diluted in 20 *μ*L reagents containing the following: 9 *μ*L MIX, 8 *μ*L H_2_O, 1 *μ*L sense primer (F), 1 *μ*L antisense primer (R), and 1 *μ*L cDNA. The same cycling parameters were repeated for 40 times. Relative content of mRNA extracted from experimental group of CA, positive control group of docetaxel, and interferon negative control group was calculated by RT-qPCR detection system BIORAD IQ5.

The article "The Studies of Chlorogenic Acid Antitumor Mechanism by Gene Chip Detection: The Immune Pathway Gene Expression" was retracted in 2020. Reason: no approval from a third party.

## 3. Results and Discussion

### 3.1. Gene Expression Profiles of Tumor Cell after Being Treated by CA

34275 probes without repeat were retained after combination and filtration. We carried out a Student's *t*-test of these probes to select differentially expressed genes (*P* ≤ 0.05) and then drew curves reflecting different expression tendency of them at 6 time points. Eighty different curves were obtained after curve fitting. The smaller the *P* value is, the more similar each gene trend fits the curve. NO.21 fitting curve had a *P* value close to 0 and the expression profiles of genes covered in this fitting curve were analyzed systematically here. As shown in Figure 1, each inflection point corresponds to gene expression at different time points after administration. Genes covered in this curve were upregulated as seen from the whole time cycle; in other word, CA is capable of upregulating certain genes of tumor-bearing mice. 

Data of genes covered in NO.21 was put into SBC Analysis System (V2010.05) and compared with KEGG (Kyoto Encyclopedia of Genes and Genomes) database. As shown in Table 2, 96 pathways are found to be related to upregulated genes and 29 of them are found to be statistically significant including T-cell receptor signaling pathway, B-cell receptor signaling pathway, and natural killer cell mediated cytotoxicity. Immune-related genes expression is speculated-changed after treatment with CA and probably have a trend of upregulation. Previous studies on CA immune function verified that CA could increase the carbon clearance index and the content of serum hemolysin and enhance the phagocytic function. Expression level of IFN-*γ* and IL-2 increased whereas that for IL-4, IL-10 decreased. The release of tumor necrosis factor (TFN) was found reduced while the activation of cytotoxic T lymphocyte (CTL) which aimed at Lewis lung cancer was boosted. NK cells activation and lymphocyte transformation rate of Lewis lung cancer bearing mice were both significantly improved through the determination of immune function indexes. To sum up, CA has been proved capable of strengthening cellular immune functions to tumor. When 3 immune related pathways were found including upregulated genes, we inferred that the immunity of mouse had been improved after treatment of CA. GSK3B, NFATC2, NFATC3, CaN, VAV2, and NCK1 were found upregulated in the 3 immune related pathways as listed in Table 3. According to the functions, genes covered in NO.21 can be classified into 312 different GO (Gene Ontology) and 6 of them has a *P* value less than 0.05 as listed in Table 4. GO of statistical significance includes the following genes: Cyp2a4, Cyp2c37, Cyp2c38, Cyp27b1, Cyp51, E4f1, Fdps, Gata4, Eif2ak1, Myt1l, Rarg, Sod1, Sp1, Taf3, Nr2c2, Hnf4g, Zdhhc3, Phf6, Mynn, Zfp386, Zfp617, Zfp114, Zfp238, Zfp174, Zfp113, Zfp109, Zfp263, Pcdhb6, Pcdhb15, Pcdhb20, Pcdhb21, Cdyl, Nfatc3, Pbx2, Rest, Smarca5, and Nfatc2. After doing some queries on the function of genes covered in statistically significant pathways and GO, we found out immune related genes and common genes of pathway and GO. Nfatc2, Nfatc3, Nfatc2ip, and CaN were found through combing raw analysis data of gene expression profile, as shown in Table 5.

The article "The Studies of Chlorogenic Acid Antitumor Mechanism by Gene Chip Detection: The Immune Pathway Gene Expression" was retracted in 2020. Reason: no approval from a third party.

### 3.2. Validation of Differentially Expressed Genes by Fluorescence Quantitative PCR

Relative expression level of the target genes Nfatc2, Nfatc3, Nfatc2ip, and CaN on average is shown in Table 6. Relative expression level of Nfatc2, Nfatc3, Nfatc2ip, and CaN in high-dose CA group, Nfatc2ip and CaN in medium-dose CA group, and CaN in low-dose CA group significantly improved compared with negative control group. The exact expression quantity is shown in Figure 2.

As shown in Figure 2, relative expression level of Nfatc2ip, Nfatc3, Nfatc2, and CaN in high-dose CA group improved compared with negative control group, which corresponds to the result of microarray analysis.

### 3.3. Discussion of Genes Nfatc2ip, Nfatc3, Nfatc2, and CaN

Here, a whole mouse genome oligo microarray (4∗44K) was used to analyze gene expression level of female BALB/c mice and to compare the expression of corresponding target genes of each group on the time series. Systematic error or accidental error can affect the accuracy of microarray analysis to some extent and the errors may come from the processes of RNA extraction, RNA reverse transcription, and hybridization as well as the quality of gene chips and RNA. While the results of microarray analysis can reflect expressing pattern at body's internal gene level quickly, false positive results possibly caused by systematic error or accidental error must be taken into consideration. Verifying experiments like ELISA test, western blot test, and PCR test should be taken for further confirmation. Here, the results of PCR test help completing the study as well as making it more convincing. Through the analysis of genes included in NO.21, expression of critical genes in T-cell receptor signaling pathway, B-cell receptor signaling pathway, and natural killer cell mediated cytotoxicity had changed and immune related genes Nfatc2ip, Nfatc3, Nfatc2, and CaN were found.

The article "The Studies of Chlorogenic Acid Antitumor Mechanism by Gene Chip Detection: The Immune Pathway Gene Expression" was retracted in 2020. Reason: no approval from a third party.

NFAT (nuclear factor of activated T cells) which consists of 4 components NFATc1, NFATc2, NFATc3, and NFATc4 has been proved important in lymphocyte activation and development. Nfatc2 existing in cytoplasm translocates to the nucleus upon T-cell receptor stimulation and then becomes a member of the nuclear factor of activating T-cells transcription [13]. When the body lacks NFATc2, lymphocyte apoptosis will be significantly reduced which suggests lymphangiectasia and Th2-type response. Meanwhile, the Th1/Th2 balance will be destroyed which suggests a Th2 polarization. Immune regulatory function will disorder when Th1/Th2 balance is destroyed and tumor occurrence shows the preponderance state tendency of Th2. This state will weaken antitumor immune function and will induce tumor cells free from immune surveillance and immune attack. This may be one of the immune mechanisms of tumor development and provides a new idea of tumor treating. The reverse of Th1/Th2 abnormal drift is in favor of recovering antitumor immunocompetence and reducing tumor recurrence and metastasis to improve long-term survival rate finally.

NFATc2 and NFATc3 have been proved to synergistically regulate the reaction of T cell receptor, cell division, and Th2 differentiation. Th2-type reaction which suggests the secretion of IL-4, IL-5, and IL-6 is increased whereas the decrease IL-2, IFN-*γ*, TNF-*α*, and IL-10 happens when the body lacks NFATc2 and NFATc3 [14–16]. When B cell and T-cell lack NFATc2 and NFATc3 simultaneously, the function of T cell will be weakened but the ability of T cell receptor mediating cell proliferation still exists, while B cells over-activate and show excessive differentiation [17]. The fact that expression of NFATc2 and NFATc3 is improved after treatment of CA indirectly indicates that CA could reverse Th1/Th2 drift. Meanwhile, secretion of IL-2, IFN-*γ*, TNF-*α*, and IL-10 is connected to CA too. High expression of NFATc2 and NFATc3 is in favor of the secretion of these cytokines which have already been used as nonspecific immunity treatment to cancer. NFATc2ip can induce the expression of T-cell cytokines, especially enhancing IL production. Three splice variants existing in NFATc2ip are able to methylate NFATc2ip after its translation to produce NFATc2ip regulatory factor. Expression of Th1-type and Th2-type cell factors will be suppressed when the methylation process is inhibited. Therefore, methylation process of NFATc2ip is an important controlling point of manipulating expression of NFAT-dependent cell factors but it will not have any influence on general transcription factor of Th1 and Th2 nor NFAT activation.

The article "The Studies of Chlorogenic Acid Antitumor Mechanism by Gene Chip Detection: The Immune Pathway Gene Expression" was retracted in 2020. Reason: no approval from a third party.

CaN (Calcineurin) is known as the only serine/threonine protein phosphatase regulated by Ca(^2+^)-calmodulin so far and mainly aims at catalyzing dephosphorylation of phosphatidylserine and phosphatidyl threonine. It is a multifunctional signaling enzyme involved in function regulation of many cells and distributes in a wide range of tissues especially nerve tissue, T lymphocytes, heart, and skeletal muscle [18, 19]. NFAT family is the main substrate of CaN. NFAT regulates many genes expression as well as influencing many cells differentiation through CaN/NFAT signaling pathway. CaN is able to make NFAT existing in cytoplasm move into cell nucleus after dephosphorylation to finish following transcription and translation, and then Nfatc can combine with AP-1 family members alone or in groups to stimulate secretion of cell factors in certain areas such as IL-2. Transcription induction of IL-2 is a sign of T-cells activation. As mentioned above, NFAT is very important in regulating immunoreaction; meanwhile, NFATc3 and NFATc2 play a particularly key role in correcting body's immune function. Thus, high expression of CaN is a benefit to dephosphorylation of NFAT and indirectly has an effect upon immune system.

## 4. Conclusion

The result of microarray analysis of differentially expressed genes of female BALB/c EMT-6 mice has indicated that the antitumor mechanism of CA is closely related to body's immune system. Through upregulating, the expression of CaN, NFATC2, NFATC2ip, and NFATC3, CA is able to improve the transcription of immune factors like IL-2R and IFN-*γ*, stimulate proliferation and activation of T cells, NK cells, and macrophage, strengthen monitoring and killing abilities of cancer cells, and inhibit growth of tumor finally. The understanding of the anticancer mechanism of CA has provided a reliable evidence of taking advantage of CA to fight against cancer.

## Figures and Tables

**Figure 1:** Expressing change of genes covered in NO.21 at 6 time points.

**Figure 2:** Relative expressing quantity of Nfatc2ip, Nfatc3, Nfatc2, and CaN in each groups. (a) Comparsion of Nfatc2ip expressing quantity among every group. (b) Comparsion of Nfatc3 expressing quantity among every group. (c) Comparsion of Nfatc2 expressing quantity among every group. (d) Comparsion of CaN expressing quantity among every groups.

**Table 1:** Primers used for RT-qPCR validation and additional expression profiling.

Gene	GenBank accession	Forward	Reverse
Nfatc3	NM_010901	CTCCCTATCATAACCCA	CTgAAggCAAATCTgTG
Nfatc2ip	NM_010900	AAAAgCAgAAAgCATACg	gACAggCCCTTCCACTA
Nfatc2	NM_010899	TgAgAAgATCgTAggCAAC	gCTCgATgTCAgCgTTT
CaN	NM_001004025	TgggAAATgAggCgATT	CCACgCTCAAAgAACCAg

The article "The Studies of Chlorogenic Acid Antitumor Mechanism by Gene Chip Detection: The Immune Pathway Gene Expression" was retracted in 2020. Reason: no approval from a third party.

**Table 2:** Pathways of upregulated genes.

Pathway name	Hits	Total	Percent (%)
Natural killer cell mediated cytotoxicity—*Mus musculus* (mouse)	4	161	2.48
B-cell receptor signaling pathway—*Mus musculus* (mouse)	5	85	5.88
T-cell receptor signaling pathway—*Mus musculus* (mouse)	6	132	4.55

**Table 3:** Upregulated genes in T-cell receptor signaling pathway, B-cell receptor signaling pathway, and natural killer cell mediated cytotoxicity.

Pathway name	GeneID	ProbeID	Symbol
Natural killer cell mediated cytotoxicity—*Mus musculus* (mouse)	18019	Nfatc2	NFATC2
	18021	Nfatc3	NFATC3
	19059	CaN	CAN
	22325	Vav2	VAV2

T-cell receptor signaling pathway—*Mus musculus* (mouse)	17973	Nck1	NCK1
	56637	Gsk3b	GSK3B
	18019	Nfatc2	NFATC2
	18021	Nfatc3	NFATC3
	19059	CaN	CAN
	22325	Vav2	VAV2

B-cell receptor signaling pathway—*Mus musculus* (mouse)	56637	Gsk3b	GSK3B
	18019	Nfatc2	NFATC2
	18021	Nfatc3	NFATC3
	19059	CaN	CAN
	22325	Vav2	VAV2

**Table 4:** GO of statistical significance.

GO ID	Name	Hits	Total	Percent (%)
GO:0009055	Electron carrier activity	7	107	6.54
GO:0003682	Chromatin binding	8	138	5.8
GO:0046906	Tetrapyrrole binding	6	107	5.61
GO:0030528	Transcription regulator activity	28	1053	2.66
GO:0009058	Biosynthetic process	73	3388	2.15
GO:0043167	Ion binding	78	3709	2.1

**Table 5:** Immune related genes covered in GO and pathway.

GenBank accession	GO ID	Gene symbol
NM_010899	GO:0001816	Nfatc2
NM_010900	GO:0001816	Nfatc2ip
NM_010901	GO:0003677	Nfatc3
NM_001004025	GO:0004723	CaN

**Table 6:** Relative expression level of target genes on average ($\overset{-}{x}\pm s$, *n* = 10).

Group	Gene			
	Nfatc2	Nfatc3	Nfatc2ip	CaN
Docetaxel	1.270 ± 1.216	1.311 ± 0.573	0.294 ± 0.160	1.136 ± 0.544
Interferon	3.831 ± 4.960	2.152 ± 1.089	0.562 ± 0.464	1.566 ± 0.914
High-dose CA	2.920 ± 2.047	4.341 ± 3.961	1.373 ± 1.096	1.961 ± 0.927
Mid-dose CA	1.086 ± 0.367	1.803 ± 1.255	0.937 ± 0.950	1.868 ± 1.160
Low-dose CA	1.185 ± 1.156	1.220 ± 1.303	0.507 ± 0.168	1.238 ± 0.310
Negative	1.085 ± 0.462	0.979 ± 0.839	0.769 ± 1.599	0.950 ± 0.418
